The article "Higher Education Environment Monitoring and Internationalization Strategy Model Using Big Data Analysis" was retracted in 2023. Reasons: unreliable results or conclusions; concerns about the data; concerns about the results or conclusions; concerns about the peer review.

# Higher Education Environment Monitoring and Internationalization Strategy Model Using Big Data Analysis

**DOI:** 10.1155/2022/4263002

**Published:** 2022-10-03

**Authors:** Minxuan Zhang

**Affiliations:** ^1^School of Education Science, Northwest Normal University, LanZhou, 730070, China; ^2^Cooperation and Exchange Office, Tianshui Normal University, Tianshui 741001, China

## Abstract

This paper creates a model based on big data, examines higher education's internationalization approach, and simultaneously conducts research. According to the research, the method used in this work has a greater accuracy rate than numerous other well-known methodologies for assessing the risk associated with higher education internationalization strategies, with the maximum accuracy rate reaching 68.9%. It can be seen that the methodology used in this report is more suited for researching the higher education sector's internationalization plan. Information integration management is advancing steadily in the age of big data. To ensure the standardization, informationalization, and scientificization of school education and teaching management, consideration should also be given to the organic integration and full utilization of education internationalization data in the field of higher education internationalization strategy.

## 1. Introduction

Higher education institutions are the practice area for internationalising higher education. At the institutional level, it is necessary to integrate and promote the development of higher education internationalization gradually. We can look at the strategic model as well as the historical and comparative perspectives as a reasonable beginning point in order to comprehend its significant implications. The globalization of higher education is both a necessity for raising educational standards in China and a strategy for the future growth of colleges and universities. Additionally, it offers a crucial assurance for the development of colleges and universities into top-tier institutions [1]. The country's goal in internationalising higher education is to raise the standard of Chinese higher education, expand its influence abroad, and develop a pool of talent with a strong sense of the global community, a broad base of knowledge, strong adaptability, and a creative spirit to meet the demands of the nation's multifaceted development. Numerous internationalization strategy models have been created as a result of the growing emphasis on the value of these models as “process” descriptions. From focusing only on academic strategy in internationalization strategy to focusing on the combination of academic strategy and organizational strategy; academic strategy is the specific content of implementation, while organizational strategy is to ensure the effective implementation of academic strategy in organization and reflect more management characteristics. First, focus on organizational structure, and then focus on the tissue process [2, 3]. Therefore, only by defining the internationalization of higher learning and understanding the differences between abilities and levels and the relationship between them can we put forward effective strategies to promote the internationalization of Chinese universities.

The article "Higher Education Environment Monitoring and Internationalization Strategy Model Using Big Data Analysis" was retracted in 2023. Reasons: unreliable results or conclusions; concerns about the data; concerns about the results or conclusions; concerns about the peer review.

Many wealthy nations have committed to the creation and use of big data in recent years and have implemented big data initiatives. China has also included big data into its national development policy in response to the promotion of big data on a worldwide scale. Realizing the fair education of the internationalization strategy of higher learning and enhancing the teaching quality of higher education depend much on how to mine the potential worth of the data and use the data information to research it [4]. Big data is quickly evolving into a new generation of information technology and service formats that gather, store, and correlate data from many different sources in various formats in order to uncover new information, create new value, and improve existing capabilities. Big data is a sort of data collection that has a high application value and is defined by its vast capacity, variety of types, and speed of access. Big data is a data set that can be processed more quickly than using conventional database systems for data collecting, storage, distribution, management, and analysis. It is the convergence of data object, technology, and application. The goal of researching the use of big data in higher education is to advance the thorough fusion of big data and higher learning internationalization strategy, effectively recognise the value of higher learning internationalization strategy data for applications, and advance the creation and revision of higher education internationalization strategy. A subset of big data is used in the internationalization strategy of higher education. It is a set of data that was created during the entire course of educational activities and gathered in accordance with educational needs. It is employed in the creation of higher education's internationalization plan and has significant potential [5, 6].

At present, the establishment of a lifelong education mechanism for teachers based on big data is a key factor in deepening the integrated development of teacher education. First of all, teachers' education experts and primary and secondary education experts should be organized to make overall design and planning for the integrated development of teacher education before and after employment and to make the integration of lifelong education mechanism concrete. In the field of higher learning, it is urgent to pay more attention to data security and data privacy protection in data management. First, establish a top-down education big data security supervision system, establish an education data security management organization, formulate data service security standards and data security management systems, and regularly conduct security audits on data [7]. Based on the analysis of big data, we will explore the regional advantages; actively serve the local political, economic, and cultural construction; actively participate in the formulation of the local government's opening-up policy and various foreign exchange activities; consciously enhance its cultural radiation function; consciously play an important role in the inheritance, development, and transmission of urban culture; assess the situation; and strive for the government's support in policy, capital, and human resources. It has promoted the pace of local high schools advancing towards the global market and improved the strength and competitiveness of the schools [8]. In the age of big data, the information integration management is becoming more and more mature. In the field of higher learning internationalization strategy, we should also pay attention to the organic integration and full utilization of education internationalization data to ensure the standardization, informatization, and scientization of school education and teaching management. Through the educational data integration information platform, the structure and functions of various departments of the school are reconstructed, and the information sources are integrated and updated, thus promoting the optimization of the international organization structure of the school.

The article "Higher Education Environment Monitoring and Internationalization Strategy Model Using Big Data Analysis" was retracted in 2023. Reasons: unreliable results or conclusions; concerns about the data; concerns about the results or conclusions; concerns about the peer review.

Under the background of big data, the international exchanges among universities in various countries are increasingly strengthened, and the forms of international cooperation are increasingly rich. In particular, there are more and more degree courses across universities, countries, and regions, and transnational and even cross regional network universities are emerging. The main contributions of this paper are as follows: (1) in this paper, the internationalization strategy model of higher learning is constructed. By using big data analysis to analyze the internal factors of the internationalization development of higher learning, we can find the advantages and disadvantages that have been held or will be faced at present, not only can we comment on the current situation of the internationalization development of higher learning but also can predict the future development situation, which is conducive to summing up the existing experience and promoting the future trend towards the goal. (2) Put up sensible initiatives and ideas to encourage the use of big data in the internationalization of higher education. Risks associated with internationalization in higher education include internationalization policy risk, internationalization development planning design and implementation risk, cooperative school risk, international student exchange risk, risk associated with bringing in foreign talent and staff training, risk associated with international academic exchange and cooperation, and risk associated with teaching reforms that are internationalization-focused.

## 2. Related Work

The idea of internationalization of higher learning has been around for a long time. However, with the development of the world today, new forms and trends have emerged in the economy, which has given the internationalization of higher learning a deeper and broader meaning and mission, and the internationalization of higher learning is gaining momentum.

Zhang and Lin put forward that the internationalization of colleges and universities involves four elements, namely, organizational change, innovation of curriculum development, development of teachers' internationalization level, and international exchange and training of students [9]. Guo and Suo show that the trend of educational globalization has made high schools gain more support from local governments. With the development of economic globalization, educational globalization has become a development trend. This provides convenience for local schools to obtain diversified investment entities, multilevel and diverse school-running patterns, and mobilize the whole society to do a good job in education [10]. Shukla and Alim reveal that the combination of offline and online teaching methods provides the possibility for the personalized development of higher learning teaching methods. Offline teaching can help students better understand and master basic theoretical knowledge, strengthen practical training, and promote the formation of students' practical knowledge [11]. Ms et al. put forward the strategy of implementing university internationalization at different levels, considering that the internationalization investment of Chinese universities can greatly promote the overall development of the society. If the limited resources of Chinese university education are wasted or put at risk, it will inevitably affect the development policy of “unifying the scale, structure, quality, and benefit” of Chinese university education [12]. Huan and Bo put forward the risks of internationalization policy of higher learning, design and implementation of internationalization development plan, cooperation in running schools, international exchange of students, introduction of foreign talents and training of teaching staff, international academic exchange and cooperation, and internationalization-oriented teaching reform [13]. Mahrous et al. show that the internationalization of colleges and universities is a development trend that includes a variety of specific activities, mainly including three aspects: first, the international content in the curriculum [14]. Chen and Tian put forward that paying attention to the international academic frontier and improving teachers' teaching and research ability and students' training quality is an important way to expand the international influence of the school and improve the internationalization level of the university. Correspondingly, teachers pay more and more attention to the important role of studying abroad in the development of the school and the improvement of their own quality [15]. Tang et al. think that the internationalization of higher learning has become a new opportunity challenge and how to evaluate the risks brought by it is of great significance and value. China's university internationalization strategy risk quantification aims at evaluating the investment risk level of the project through the evaluation of risk interaction, so as to determine the feasibility and value of the project [16]. Zhaoheng believes that in the process of internationalization, colleges and universities generally send students and teachers to overseas schools to study or engage in scientific research, thus promoting exchanges between schools and maximizing the scientific research strength of local universities [17]. Chen et al. show that in order to better meet the needs of economic and social development, especially the opening-up to the outside world, many local high schools have set up characteristic majors and applied majors that are easy to be in line with international standards and in line with their own development on the basis of building their original majors [18].

The article "Higher Education Environment Monitoring and Internationalization Strategy Model Using Big Data Analysis" was retracted in 2023. Reasons: unreliable results or conclusions; concerns about the data; concerns about the results or conclusions; concerns about the peer review.

In view of the research made by previous scholars, this paper studies the internationalization strategy of higher learning based on big data analysis and builds a model. Establishing the risk assessment index system of internationalization strategy of Chinese universities is the basis of risk assessment of internationalization strategy of Chinese universities. Analytic hierarchy process (AHP) is used to synthesize indicators based on big data analysis, which involves many qualitative evaluation indicators. The weight of each indicator is the basic parameter of the evaluation system, and the qualitative data must be processed in the process of its determination. When we focus on using the internationalization of higher learning to obtain economic benefits, the geographical relationship can only play a certain role in promoting it, because whether our own higher learning strength has global competitiveness is the key to obtain economic benefits. In combination with reality, special attention should be paid to learning from the school-running characteristics and successful management experience of foreign educational institutions, so that educational institutions can truly have comparative advantages. Based on big data analysis, we will introduce foreign high-quality educational resources to optimize and integrate the existing teaching resources and make the internationalization of higher learning more dynamic and vigorous.

## 3. Research Method

### 3.1. Construction of Internationalization Model of Higher Education Based on Big Data

At present, there are many theories on the definition of the connotation of the internationalization of higher learning in the academic circles of various countries. The “result theory” theory represented by the Japanese scholar Yoshimura believes that the internationalization of higher learning means that the national culture is recognized and accepted by other countries and nations and has received appropriate evaluation [19]. The internationalization of higher learning is actually to be in the international higher learning environment and compete with the higher learning of other countries in the world. Before formulating the higher learning strategy, we must make a correct analysis of the advantages and disadvantages of higher learning itself and its opportunities and threats in the international environment and make a correct understanding of the current situation of higher learning internationalization, so as to judge what advantages higher learning can play in the process of internationalization. What disadvantages need to be improved, and what opportunities and threats will there be in the process.

The school should try its best to create conditions for students so that they can have more opportunities to contact with foreign cultures. This not only requires teachers to introduce the latest research trends and achievements in the world in the classroom but also provides possible conditional support for teachers and students [20]. It is true that the international academic community has a common view on the internationalization of higher learning, whether it is the “result theory” and “process theory” or the “macro round” and “micro round”. They unanimously believe that the internationalization of higher learning refers to the process of cross-country and cross regional exchanges and cooperation of higher learning in this region; many higher learning factors in this region, including modes and concepts, should be recognized and accepted by other countries or regions and the specific process and activities of actual communication with other target countries or regions. Based on big data analysis, this paper builds the strategy model of higher learning internationalization and analyzes the four macro factors such as politics, economy, society, and technology that affect the development of higher learning internationalization by using the analysis model, which is conducive to approaching the strategic height and looking at the development of higher learning internationalization from the overall perspective. The internationalization strategy model of higher learning is shown in Figure 1.

The article "Higher Education Environment Monitoring and Internationalization Strategy Model Using Big Data Analysis" was retracted in 2023. Reasons: unreliable results or conclusions; concerns about the data; concerns about the results or conclusions; concerns about the peer review.

Big data analysis can be used to identify the benefits and drawbacks that have been experienced or will be felt in the near future when internal elements of higher education's internationalization are examined. It can make observations about how higher education is developing internationally as well as make predictions about what will happen in the future, which helps to summarise past experience and encourage future trends in the direction of the objective [21]. According to the characteristics of the research data, the bell-shaped membership function is used as the variable fuzzification function. Specifically, it is defined as let a fuzzy quantity be determined by *a*, *b*, and *c* and have a bell-shaped membership function.

(1) $$\begin{array}{c} \mu \left(x\right)=\left[\frac{1}{1+\left(\left(x-c\right)/\alpha \right)}\right]. \end{array}$$

Where *a* represents the deviation coefficient of the fuzzy quantity, which reflects the numerical divergence of the fuzzy quantity.

Thereby forming an initial evaluation matrix *R*.

(2) $$\begin{array}{c} R=\left[\begin{array}{c} \left[a_{11},b_{11},c_{11}\right]\\ \left[a_{p1},b_{p1},c_{p1}\right] \end{array}\right]. \end{array}$$

Thereby, forming a weight set of expert evaluation.

(3) $$\begin{array}{c} E=\left[e_{1}\cdots e_{p}\right]. \end{array}$$

Therefore, this operator is used for fuzzy synthesis, thus forming a fuzzy synthesis matrix.

(4) $$\begin{array}{c} F=〚a_{1}\;b_{1}\;c_{1}〛. \end{array}$$

According to the bell-shaped fuzzy quantity calculation formula, the fuzzy weight of the *i* index is

(5) $$\begin{array}{c} \tau_{i}=2b+c_{i}. \end{array}$$

And the fuzzy weight set is obtained after normalization.

(6) $$\begin{array}{c} W_{\tau }=\left\lfloor \begin{array}{cccc} \tau_{1} & \tau_{2} & \cdots & \tau_{p} \end{array}\right\rfloor . \end{array}$$

The entropy of fuzzy event *A* is defined as

(7) $$\begin{array}{c} H\left(A\right)=-\overset{n}{\underset{i=1}{\sum }}\mu_{A}P_{i}\ln P_{i}. \end{array}$$

Where *A* is the fuzzy event in {*x*_1_, *x*_2_, ⋯*x*_*n*_}.

The article "Higher Education Environment Monitoring and Internationalization Strategy Model Using Big Data Analysis" was retracted in 2023. Reasons: unreliable results or conclusions; concerns about the data; concerns about the results or conclusions; concerns about the peer review.

Based on the above definition, the fuzzy entropy evaluation model of internationalization strategy risk of higher learning can be expressed as follows

(8) $$\begin{array}{c} H\left(A\right)=-\overset{n}{\underset{i=1}{\sum }}K\left({\alpha \mu }_{A}\left(x_{i}\right)\right). \end{array}$$

When *α* = 1, the generalized entropy of fuzzy event *A* in the strategic risk of internationalization of higher learning becomes the entropy definition of fuzzy event *A*.

On the basis of fuzzy matrix *R* of bell-shaped membership function, the total entropy of the *i* index is determined to be

(9) $$\begin{array}{c} H_{i}=-\frac{1}{31nn}\underset{a,b}{\sum }. \end{array}$$

In the formula, the meaning of *a*, *b* is as described above.

On the basis of the index total entropy formula, calculate the *i* index entropy weight as follows:

(10) $$\begin{array}{c} \rho_{i}=\left(\frac{H_{i}}{\sum_{i=1}^{p}H_{i}}\right). \end{array}$$

Thus, the entropy weight set is obtained.

In this sense, the internationalization of higher learning should be a dynamic development process. However, for the edge/center dimension of higher learning internationalization, it is difficult to evaluate it only according to the literature. Even if the evaluation is a subjective evaluation, it lacks obvious quantifiable indicators.

Big data analysis of the globalization of higher education has revealed the necessity to construct a global education paradigm in line with the demands of contemporary growth. Only in this way, based on big data analysis, can colleges and universities run their schools in a self-aware and purposeful manner, enabling international education to be self-aware and purposeful in general behaviour and facilitating the rapid growth of the internationalization of higher learning [22]. We actively support the education of international students through the study of large amounts of data. Colleges and universities have put a lot of effort into international exchange and collaboration, the training of instructors abroad, the education of international students, the employment of foreign teachers, and overseas exchange programmes. These initiatives have helped to increase the degree and popularity of globalization of higher education while also somewhat speeding up its development.

The article "Higher Education Environment Monitoring and Internationalization Strategy Model Using Big Data Analysis" was retracted in 2023. Reasons: unreliable results or conclusions; concerns about the data; concerns about the results or conclusions; concerns about the peer review.

### 3.2. Suggestions on Measures to Promote Big Data Application in Internationalization Strategy of Higher Education

The internationalization of colleges and universities involves four elements: organizational change, innovation of curriculum development, development of teachers' internationalization level, and international exchange and cultivation of students. There is a special interdependence and mutual restriction relationship between economy and education. When economic globalization has become a reality and necessity, it is bound to have a profound and extensive impact on education, which will inevitably lead to more frequent exchanges and cooperation of educational resources in the world, and at the same time, force the educational resources of various countries to open to the world [23]. In the rapidly changing process of international social and economic development, in order to maintain its competitiveness, the university system must always face challenges and opportunities. Starting from the needs of social and economic development, we should seek to improve the internationalization level of university organization, curriculum innovation, teacher development, and student training.

Managers and staff members involved in transnational operations should be knowledgeable with local politics, economics, and culture in addition to the laws of international economic operation. Under the trend of economic globalization, this is the fundamental prerequisite for talents to carry out international operations and collaboration. The objective demand of the market, which is an unavoidable trend regardless of human volition, has encouraged the internationalization of education. Risks of higher learning internationalization policy, design and implementation of internationalization development planning, cooperation in running schools, international exchange of students, introduction of foreign talents and training of teaching staff, international academic exchange and cooperation, and internationalization-oriented teaching reform. The risk evaluation index system of higher learning internationalization strategy is represented as a hierarchical structure, as shown in Figure 2.

The promotion of the use of big data in higher education needs to start from the following aspects in light of the issues with inadequate technology, a solitary data island, a lack of professionals, and ineffective laws and regulations in the application of big data in China's higher education's internationalization strategy.

#### 3.2.1. Attach Importance to the Training of Professionals and Improve the Quality of Data Services

Colleges and universities should change the composition of teaching and administrative teams, enhance post settings, and actively recruit individuals with skills in big data management and application. In light of this, higher education's internationalization strategy must fully take into account the Internet's contribution to the growth of educational and teaching activities, fully utilise big data technology for data collection and statistical analysis, and view the Internet and big data as significant teaching resources. Schools can better comprehend future directions and the focus of professional education by using education and teaching as a source of information and raw materials.

The article "Higher Education Environment Monitoring and Internationalization Strategy Model Using Big Data Analysis" was retracted in 2023. Reasons: unreliable results or conclusions; concerns about the data; concerns about the results or conclusions; concerns about the peer review.

#### 3.2.2. Unify Data Caliber and Build a Big Data Platform

By creating a big data platform, you may more effectively mine a variety of data sources and create the groundwork for integrating, analysing, and sharing big data. The information flow in the network environment is what creates the data. These data will be gathered during this process and used to meet the audience's specific needs and improve the services being offered to them.

#### 3.2.3. Strengthen Policy Guidance and Promote the Benign Development of Big Data in Higher Learning

Higher education's use of big data has also contributed to advancements in auxiliary management, precision teaching, tailored learning, and educational equity. Naturally, there are a lot of issues as well, like data ownership, data privacy, and data security. Higher education's internationalization plan activities generate a significant amount of audio and video data, primarily in the form of activity and course videos. Although they will take up a lot of room, this informational data can be employed as significant instructional materials. In order to meet the actual needs of data storage in colleges and universities, it is important to further improve the data information storage within the lower cost limit.

The management work in the process of internationalization is a systematic, targeted, planned, and relatively complete institutional process. The internationalization strategy of colleges and universities clarifies the meaning of the internationalization of colleges and universities and the specific work to be undertaken—formulate specific medium- and long-term goals to ensure the orderly implementation of the internationalization work and train teachers, analyze cost-effectiveness, etc. The construction of the big data platform for the internationalization strategy of colleges and universities needs to break the original situation of each department fighting its own way; carry out the automatic collection and storage of information data in colleges and universities; comprehensively carry out the construction of office automation in colleges and universities; further upgrade and optimize the collection, storage, and management system of financial management data; and carry out international strategy teaching information management and teaching quality inspection.

The article "Higher Education Environment Monitoring and Internationalization Strategy Model Using Big Data Analysis" was retracted in 2023. Reasons: unreliable results or conclusions; concerns about the data; concerns about the results or conclusions; concerns about the peer review.

## 4. Analysis and Discussion of Results

This paper only analyzes the four provinces of Beijing, Shanghai, Gansu, and Shaanxi, which use their geographical advantages to recruit international students for key partners. According to Table 1, “Number of students in colleges and universities per 100,000 population,” the development level of higher learning in Gansu and Shaanxi is in the downstream position, ranking third and fourth, respectively.

By opening up a “University City,” building five higher learning parks, and encouraging social forces to participate in higher learning and other measures, this experiment has rapidly expanded the scale of higher learning in Zhejiang Province in a short period of time, creating a miracle year. The college entrance examination admission rate (a) is as high, and the gross enrollment rate (b) of higher learning reaches the internationally accepted starting point goal of higher learning popularization for the first and the average gross enrollment rate of higher learning can reach 25.5%. The gross enrollment rate of higher learning in the country increased to more than 25.5% from 2018 to 2021, and the gross enrollment rate of higher learning exceeded the national average. The admission rate of business examination and the gross enrollment rate of higher learning in 2012-2021 are shown in Figure 3.

During this period, the number of college enrollment, students, and graduates also increased greatly. As shown in Figure 4, the average number of graduate enrollment is about 6,416, the number of students is about 8,079, and the number of graduates is about 4,200. As shown in Figure 5, the average enrollment of graduate students in this college is about 171,529, the number of students in school is about 412,948, and the number of graduates is about 85,230. However, because of the rapid growth, the rapid expansion of enrollment in Zhejiang Province also brings a series of problems such as the decline of education quality and employment.

The analysis and evaluation of China's education opening to the outside world and international development, a cooperative project of the International Education Exchange Association and Shanghai Jiao Tong University, is a version of the “Questionnaire of Education Opening in Provincial Administrative Regions” designed by the research group, which involves the distribution of overseas students in different countries and regions. The questionnaire was filled in through the online filling system of China's universities' international development survey. The questionnaire was distributed to all universities with undergraduate level in Gansu, Shaanxi, and Shanghai. There were 63 universities in three provinces, and 63 questionnaires were distributed. From April 17th, 2022 to June 28th, 2022, a total of 15 valid questionnaires were collected, with a recovery rate of 20%. The university departments that filled in the questionnaire included International Exchange and Cooperation Office and Academic Affairs Office, as shown in Table 2.

The article "Higher Education Environment Monitoring and Internationalization Strategy Model Using Big Data Analysis" was retracted in 2023. Reasons: unreliable results or conclusions; concerns about the data; concerns about the results or conclusions; concerns about the peer review.

In addition, according to the classification of colleges and universities with the right to grant doctoral and master's degrees and ordinary undergraduate colleges and universities, it can be found that the samples participating in the questionnaire are mainly those with the right to grant doctoral and master's degrees, accounting for 71.17%, as shown in Table 3.

The basic function of a university is to cultivate talents. A good university must have a good talent cultivation ability. In the era of globalization, students can move around the world. A good university can attract international students from all over the world, which is yearned for by international students. Therefore, the proportion of international students can be a good measure of a university's talent cultivation ability. In this experiment, the proportion of international students among graduate students in world-class universities and Zhejiang University in 2021 was studied. Harvard University, Oxford University, and The University of Tokyo were used for the experiment, and the experimental results are shown in Figure 6.

It can be seen from Figure 6 that the education of international students is important to colleges and universities. At present, many colleges and universities have formulated some measures to attract foreign students and Hong Kong and Macao students. However, because the overall level of teachers is relatively poor, apart from some advantageous majors, they are not very attractive to overseas students, and the proportion of overseas students is still very low.

Finally, this experiment analyzes the accuracy rate of the internationalization strategy risk of higher learning through three methods, using the method in literature [6], literature [15], and the method in this paper. The experimental results are shown in Figure 7.

The data in Figure 7 above show that, of the three methods, the method used in this paper has the highest accuracy rate in terms of the risk of higher education's internationalization strategy, with the highest accuracy rate reaching 68.9%. The method in literature [6] is the second most accurate method. The highest accuracy rate, according to the statistics, can also reach 56.4%, and the approach described in literature [15] has the lowest accuracy rate, at only 47.8%. It can be seen that the methodology used in this work is more suited for the investigation of higher education's internationalization plan.

The article "Higher Education Environment Monitoring and Internationalization Strategy Model Using Big Data Analysis" was retracted in 2023. Reasons: unreliable results or conclusions; concerns about the data; concerns about the results or conclusions; concerns about the peer review.

## 5. Conclusion

The internationalization of higher learning is an inevitable trend of the development of higher learning. As a developing country, the development history of China's higher learning internationalization is not long and the scale is not large. Colleges and universities rarely have the opportunity to participate in the formulation of the rules of higher learning internationalization. Therefore, it is the mission of Chinese colleges and universities to transform passivity into initiative to meet the challenges of higher learning internationalization. This paper analyzes the internationalization strategy of higher learning based on big data, builds a model, and conducts research at the same time. The research shows that the accuracy rate of the method adopted in this paper in the risk of internationalization strategy of higher learning is the highest, with the highest accuracy rate reaching 68.9%, followed by the method in literature [6]. According to the data, the highest accuracy rate can also reach 56.4%, and finally the method in literature [15], with the highest accuracy rate of only 47.8%. It can be found that the method adopted in this paper is more suitable for the study of the internationalization strategy of higher learning. In the process of coping with internationalization, Chinese universities have adopted various strategies through big data analysis. What are the advantages and disadvantages of these strategies in the implementation process, what needs to be improved, and what needs to be supplemented or adjusted in the face of the constantly developing situation in the future? Through the analysis of big data, the internationalization of higher learning has also expanded the development space of higher learning and enabled higher learning to integrate into the international community. Seizing these opportunities, the international competitiveness of higher learning will be greatly improved.

## Figures and Tables

**Figure 1:** Strategic model of internationalization of higher learning.

**Figure 2:** Risk evaluation index system of internationalization strategy of higher learning.

**Figure 3:** Admission rate of business examination and gross enrollment rate of higher learning in 2012-2021.

The article "Higher Education Environment Monitoring and Internationalization Strategy Model Using Big Data Analysis" was retracted in 2023. Reasons: unreliable results or conclusions; concerns about the data; concerns about the results or conclusions; concerns about the peer review.

**Figure 4:** Number of graduate students in 2012-2021.

**Figure 5:** Number of college students in 2012-2021.

**Figure 6:** Proportion of international students in world-class universities in 2021.

**Figure 7:** Accuracy rate of internationalization strategy risk of higher learning.

**Table 1:** Ranking of the number of students and the proportion of foreign students in the number of students.

Country/province	Ranking of students in colleges and universities	Number of college students	Ranking of international students in the number of students	Proportion of international students in the number of students
Beijing	1	5471	2	1.43%
Shanghai	2	3425	1	5.48%
Guangxi	3	1940	4	1.11%
Yunnan	4	1662	3	1.19%

**Table 2:** Basic information of questionnaire distribution and recovery.

Province	Number of questionnaires issued	Number of returned questionnaires	Questionnaire recovery rate
Shanghai	25	3	8.34%
Guangxi	24	9	34.79%
Yunnan	14	3	15.39%
Total	63	15	20%

**Table 3:** Levels and categories of universities where questionnaires are issued and universities where questionnaires are valid.

Province	Colleges and universities	Proportion of universities with the right to confer doctoral and master's degrees	Proportion of undergraduate colleges and universities
Shanghai Guangxi	Questionnaire distribution colleges and universities	69.24%	30.78%
	Effective questionnaire colleges and universities	100%	0
Yunnan Shanghai	Questionnaire distribution colleges and universities	45.84%	54.18%
	Effective questionnaire colleges and universities	51%	52%
Guangxi	Questionnaire distribution colleges and universities	47.84%	52.18%
	Effective questionnaire colleges and universities	62.51%	37.52%
Total	Questionnaire distribution colleges and universities	54.30%	45.71%
	Effective questionnaire colleges and universities	71.17%	29.84%

## Data Availability

The data used to support the findings of this study are available from the corresponding author upon request.
